# Automatic Assessment of Mitral Regurgitation Severity Using the Mask R-CNN Algorithm with Color Doppler Echocardiography Images

**DOI:** 10.1155/2021/2602688

**Published:** 2021-09-13

**Authors:** Qinglu Zhang, Yuanqin Liu, Jia Mi, Xing Wang, Xia Liu, Fenfen Zhao, Cuihuan Xie, Peipei Cui, Qingling Zhang, Xiangming Zhu

**Affiliations:** ^1^Anhui Provincial Hospital, Cheeloo College of Medicine, Shandong University, Jinan, Shandong 250012, China; ^2^Department of Special Examination, Shandong Provincial Third Hospital, Cheeloo College of Medicine, Shandong University, Jinan, Shandong 250031, China; ^3^Department of Ultrasound, The First Affiliated Hospital of Wannan Medical College, Wuhu, Anhui 241001, China; ^4^Department of Neurosurgery, The First Affiliated Hospital of Shandong First Medical University, Jinan, Shandong 250014, China; ^5^Anhui Provincial Hospital, Hefei, Anhui 230001, China

## Abstract

Accurate assessment of mitral regurgitation (MR) severity is critical in clinical diagnosis and treatment. No single echocardiographic method has been recommended for MR quantification thus far. We sought to define the feasibility and accuracy of the mask regions with a convolutional neural network (Mask R-CNN) algorithm in the automatic qualitative evaluation of MR using color Doppler echocardiography images. The authors collected 1132 cases of MR from hospital A and 295 cases of MR from hospital B and divided them into the following four types according to the 2017 American Society of Echocardiography (ASE) guidelines: grade I (mild), grade II (moderate), grade III (moderate), and grade IV (severe). Both grade II and grade III are moderate. After image marking with the LabelMe software, a method using the Mask R-CNN algorithm based on deep learning (DL) was used to evaluate MR severity. We used the data from hospital A to build the artificial intelligence (AI) model and conduct internal verification, and we used the data from hospital B for external verification. According to severity, the accuracy of classification was 0.90, 0.89, and 0.91 for mild, moderate, and severe MR, respectively. The Macro F1 and Micro F1 coefficients were 0.91 and 0.92, respectively. According to grading, the accuracy of classification was 0.90, 0.87, 0.81, and 0.91 for grade I, grade II, grade III, and grade IV, respectively. The Macro F1 and Micro F1 coefficients were 0.89 and 0.89, respectively. Automatic assessment of MR severity is feasible with the Mask R-CNN algorithm and color Doppler electrocardiography images collected in accordance with the 2017 ASE guidelines, and the model demonstrates reasonable performance and provides reliable qualitative results for MR severity.

## 1. Introduction

Mitral regurgitation (MR) is a common valvular heart condition. A study by the 2016 American Heart Association (AHA) in the USA estimated that the incidence rate of moderate or worse MR is 1.7%, which is approximately 4-fold higher than that of aortic stenosis [1]. Furthermore, the incidence increases with age, and the proportion can reach 10% in the population over 75 years old [2]. The therapeutic method varies based on the degree of MR. According to the Society of Thoracic Surgeons national database, the number of mitral valve surgeries increased by an average of 4% every year between 2010 and 2015. When deciding which patients are suitable for mitral valve (MV) surgery, the guidelines of the American College of Cardiology (ACC) and AHA for the management of valvular heart disease emphasize the severity of MR [3]. Thus, accurate assessment of MR severity is crucial for clinical decision-making, prognostication, and decisions regarding the timing of surgical intervention [4]. Transthoracic echocardiography (TTE) is the most important imaging method for MR diagnosis and evaluation due to its widespread availability, low cost, acceptability, and safety profile [5]. However, the MR evaluation parameters listed in the 2017 American Society of Echocardiography (ASE) guidelines are numerous and complex and are very challenging to use in practice [6]. There is currently no single recommended MR evaluation method in this setting. Herein, we attempt to validate a convenient and automatic method for evaluating MR severity.

Since John MacCarthy first proposed “artificial intelligence (AI)” in 1956, researchers have made great efforts to apply AI to almost all stages of clinical practice. At present, the development of AI in the field of ultrasound medicine to improve the accuracy of ultrasound diagnosis, reduce the misdiagnosis rate, and meet growing clinical needs is a hot research topic. Deep learning (DL) is a subset of AI inspired by the workings of the human brain, commonly referred to as an artificial neural network (ANN) [7]. Convolutional neural networks (CNNs) are a subtype of ANNs that mimic the visual cortex. Regions with CNN features (R-CNN) apply CNNs in object detection. To improve efficiency, Fast R-CNN combines the feature extraction, classification, and bounding box prediction of R-CNN and incorporates a method called region of interest pooling (RoIPool) [8]. Then, researchers developed Faster R-CNN, which has similar accuracy to Fast R-CNN, but the training time and testing time are 10 times shorter. He et al. proposed a new method called Mask R-CNN in 2017, which expands Faster R-CNN by adding branches used to predict the segmentation mask on each of the RoIs classified with existing branches and border frame returns [9]. Compared to Faster R-CNN, the mask branch only adds a small computational overhead, enabling a fast system and rapid experimentation. Thus, our study chose Mask R-CNN algorithm. Such an AI system has great potential for effective improvement of diagnosis.

We aimed to evaluate the feasibility and accuracy of MR severity detection with AI data models using MR color Doppler echocardiography images collected based on the 2017 ASE guidelines.

## 2. Methods

### 2.1. Establishment of the MR Color Doppler Echocardiography Case Database

#### 2.1.1. Ultrasound Instrument

Ultrasound was performed by echocardiographers using a Philips ultrasound machine (EPIQ 7C, Philips Medical Systems, Bothell, WA), GE ultrasound machine (VIVID E95, GE Medical Systems, Horten, Norway), and Siemens ultrasound machine (SC2000, Siemens Medical Solutions USA, Inc.).

#### 2.1.2. Patients and MR Image Classification Standard

This study involved data from two large general hospitals in different regions. Hospital A is Shandong Provincial Third Hospital, and hospital B is The First Affiliated Hospital of Wannan Medical College. The Institutional Review Boards of the two hospitals approved this study protocol and waived the need for informed consent due to a minimal potential for harm.

All echocardiographers were well experienced, had worked more than five years, and had undergone thorough professional training before the study. According to the quantitative methods of MR evaluation from the 2017 ASE guidelines (see Figure 1), the severity of MR can be classified into three types: mild, moderate, and severe. This classification is relatively broad and cannot well reflect the severity of MR. Then, MR was further subclassified into four grades: grade I (mild), grade II (moderate), grade III (moderate), and grade IV (severe). A total of 1132 and 295 MR cases were collected from hospital A and hospital B, respectively, from January 2019 to December 2020. There were a similar number of cases for each grade. The 2017 ASE guidelines provide distinct criteria for the classification of chronic MR using color Doppler echocardiography: vena contracta (VC), effective regurgitant orifice (ERO), regurgitant volume (RVol), and regurgitation fraction (RF) [6]. VC is a parameter used for determination of the regurgitant orifice. To obtain the VC, we measure the narrowest width of the jet as it emerges from the orifice in zoom mode on the long axis view of the sternum. When determining the ERO, it is important to carefully measure the proximal isovelocity surface area (PISA) and obtain the greatest PISA radius at the time of peak MR velocity. To obtain the most hemispheric flow convergence, we adjust the lower Nyquist limit to 30-40 cm/sec. The Nyquist limit should be set at 50-70 cm/sec when measuring RF. RVol is measured in the case of multiple jets or eccentric jets, as it is more accurate. Color Doppler echocardiography images are acquired from the standard two-dimensional (2D) apical 4-chamber view of TTE or the standard view with the most regurgitation.

#### 2.1.3. Exclusion Criteria

Cases were excluded if the image quality was very poor or TTE images could not be clearly displayed.

### 2.2. Image Marking

The LabelMe software (3.167) was used to demarcate the region of interest (RoI) in MR ultrasound images for automatic analysis by machine DL technology. The workflow of LabelMe is shown in Figure 2. At the “Annotation” step, tracing the contour of MR, the more accurate the better (see Figure 3).

### 2.3. Establishment and Validation of the Data Model

#### 2.3.1. Network Architecture

Mask R-CNN is a method of object detection and segmentation that can distinguish different objects in images and draw bounding boxes (bbox) around specific objects. It can also mark and classify targets and identify other detection key points. The network architecture was constructed in the Google TensorFlow framework, and the network architecture of the Mask R-CNN algorithm is illustrated in Figure 4. We defined a multitask loss on each sampled RoI as *L* = *L*_cls_ + *L*_bbox_ + *L*_mask_. The classification loss (*L*_cls_) and bounding box loss (*L*_bbox_) were identical to those defined in Faster R-CNN [8].

(1) $$\begin{array}{c} L_{\text{cls}}=\frac{1}{N_{\text{cls}}}\underset{\text{ⅈ}}{\sum }L_{\text{cls}}\left(p\text{i},p_{\text{i}}^{*}\right), \end{array}$$

(2) $$\begin{array}{c} L_{\text{bbox}}=\frac{1}{N_{\text{box}}}\underset{\text{ⅈ}}{\sum }p_{\text{i}}^{*}L_{1}^{\text{smooth}}\left(t\text{i}–t_{\text{i}}^{*}\right), \end{array}$$

(3) $$\begin{array}{c} L_{\text{cls}}\left(\left\{p\text{i},p_{\text{i}}^{*}\right\}\right)=–p_{\text{i}}^{*}\log p_{\text{i}}^{*}-\left(1-p_{\text{i}}^{*}\right)\log\left(1-p_{\text{i}}^{*}\right). \end{array}$$

*L*_mask_ is the average binary cross-entropy loss.

(4) $$\begin{array}{c} L_{\text{mask}}=–\frac{1}{m^{2}}\underset{1≦\text{ⅈ}\leq m}{\sum }\;\left[y_{ij}\log oy_{\text{ⅈ}j}^{k}+\left(1-y_{\text{ⅈ}j}^{k}\right)\log\left(1-oy_{\text{ⅈ}j}^{k}\right)\right]. \end{array}$$

The loss function value (*L*), *L*_cls_ + *L*_bbox_ + *L*_mask_, in the Mask R-CNN was minimized.

#### 2.3.2. Network Training and Testing

The Mask R-CNN was trained using the MR ultrasound images. The MR images acquired from hospital A made up dataset A, and the MR images acquired from hospital B made up dataset B. Dataset A was used for training of the AI model. To ensure the accuracy and stability of the model, we used dataset B to verify the model. The ratio of dataset A to dataset B is approximately 8 : 2. The ratio of each grade in the two datasets is also approximately 8 : 2. The trained model was applied for prediction in the test set. The training parameters were set as follows: For the backbone and region proposal network (RPN), learning rate was 0.001; for the R-CNN and Mask heads, learning rate was 0.0001. Throughout the training process, the momentum was set to 0.9 and the stochastic gradient descent optimizer was used. The learning rate and momentum were set by monitoring the loss during training. With a low learning rate, the improvements will be linear.

#### 2.3.3. Evaluation Metrics

The overall performance of the AI model for the assessment of MR severity was validated with accuracy, precision, recall, F1-score, Macro F1, and Micro F1.

Accuracy is the ratio of the number of examples consistent with the results of the 2017 ASE guidelines and the total number of examples.

(5) $$\begin{array}{c} \text{Precision}=\frac{\text{TP}}{\text{TP}+\text{FP}}, \end{array}$$

(6) $$\begin{array}{c} \text{Recall}=\frac{\text{TP}}{\text{TP}+\text{FN}}, \end{array}$$

(7) $$\begin{array}{c} \text{F}1-\text{score}=\frac{2*\text{precision}*\text{recall}}{\text{precision}+\text{recall}}. \end{array}$$

*Macro F1*. Split the evaluations of *n* categories into *n* two-category evaluations, calculate the F1-score of each two-category, and the average value of the n F1-scores is Macro F1.

*Micro F1*. Divide the evaluations of n categories into *n* two-category evaluations, and add the corresponding TP, FP, and RN of the *n* two-category evaluations to calculate the precision and recall. The F1-score calculated from these precision and recall is Micro F1.

TP is the number of true positives, FP is the number of false positives, and FN is the number of false negatives.

## 3. Results

In this study, 1132 MR ultrasound images (288 grade I, 278 grade II, 270 grade III, and 296 grade IV) in dataset A and 295 MR ultrasound images (82 grade I, 75 grade II, 74 grade III, and 64 grade IV) in dataset B were finally applied. The baseline demographic and TTE characteristics of the study patients are summarized in Table 1.

Figure 5 shows the model performance evaluation metrics and results. The total loss was 0.0493, the bbox loss was 0.0055, the class loss was 0.0012, and the mask loss was 0.0427.

Figure 6 shows four test examples for the assessment of MR severity. Figures 6(a)–6(d) are graded MR images obtained by the evaluation methods described in the 2017 ASE guidelines. Figures 6(e)–6(h) are the results of the test using this AI model, which are consistent with the results obtained by the evaluation methods described in the 2017 ASE guidelines.

Figure 7 shows the confusion matrix of the MR classification and grading results for the validation. The accuracy of classification according to severity was 0.90, 0.89, and 0.91 for mild, moderate, and severe MR, respectively. The accuracy of classification according to grade was 0.90, 0.87, 0.81, and 0.91 for grade I, grade II, grade III, and grade IV, respectively.

Figure 8 shows the comparative histograms of precision, recall, and F1-score between classification indexes (Figure 8(a) is the classification according to severity, and Figure 8(b) is the classification according to grading). The precision of classification according to severity was 0.94, 0.93, and 0.87 for mild, moderate, and severe MR, respectively. The precision of classification according to grade was 0.94, 0.88, 0.88, and 0.87 for grade I, grade II, grade III, and grade IV, respectively. The recall of classification according to severity was 0.94, 0.90, and 0.92 for mild, moderate, and severe MR, respectively. The recall of classification according to grade was 0.94, 0.89, 0.82, and 0.92 for grade I, grade II, grade III, and grade IV, respectively. The F1-score of classification according to severity was 0.94, 0.91, and 0.89 for mild, moderate, and severe MR, respectively. The F1-score of classification according to grade was 0.94, 0.88, 0.85, and 0.89 for grade I, grade II, grade III, and grade IV, respectively. It can be observed that this model produces satisfactory precision, recall, and F1-score results in the evaluation of MR severity.

Table 2 shows the comparison results of Macro F1 and Micro F1 in each classification. This shows a satisfactory classification result.

## 4. Discussion

We validated the Mask R-CNN algorithm for the evaluation of MR severity. The present study demonstrated the feasibility and accuracy of the Mask R-CNN algorithm for qualitative assessment of MR and demonstrated the reasonable performance of the model.

TTE is the most common imaging technique by which MR severity and etiology are determined. Although many recent studies have shown that 2D technology is not the most accurate method for quantitatively evaluating MR, the 2D TTE technique is currently the most commonly used method for quantitatively evaluating MR compared with cardiac magnetic resonance (CMR), transesophageal echocardiography (TEE), and the 3D TTE technique [10]. However, there is currently no single echocardiographic parameter that is precise enough to quantify MR. Integration of multiple parameters is required for a more accurate assessment of MR severity [11]. When multiple parameters are concordant, MR severity, especially mild and severe MR, can be determined with high confidence. In our study, all MR grades were determined independently by two well-experienced echocardiographers according to the 2017 ASE guidelines. It is necessary to emphasize that when there is consistent evidence from different parameters, it is easy to grade MR severity with confidence. When different parameters are contradictory, one must look carefully for technical and physiologic factors to explain the discrepancies and repeat the measurements according to the 2017 ASE guidelines. If the discrepancy remained, a third investigator's recommendation was used as a reference. Errors in measurement can be prevented.

AI is a powerful technological driving force at present. Increasing efforts have been made by medical ultrasound experts, mathematicians, and computer scientists to promote the integration of ultrasound, medicine, and AI, thereby improving the accuracy of ultrasonic diagnosis, reducing the misdiagnosis rate, shortening the reporting time, and meeting growing clinical needs [12].

AI has made some progress in the assessment of MR; here, we review some recent studies. Many studies of MR diagnosis have been carried out to investigate heart sounds (HSs). Maglogiannis et al. used Doppler heart sound (DHS) data with wavelet decomposition followed by a three-step diagnosis phase based on support vector machine (SVM) classifier to classify heart valve disease. The reported accuracy for aortic stenosis (AS) and MR classification is 91.67% [13]. Safara et al. developed a multilevel basis selection (MLBS) method with an SVM classifier to classify normal AS MR and AR samples, and the accuracy of classification was 97.56% [14]. There are some other AI studies on the detection of MR. An intelligent diagnostic system based on automatic diagnostic feature extraction for diagnosing heart diseases developed by Sun could discriminate MR with an accuracy of 98.4% [15]. Kwon, MD, and colleagues developed and validated an AI algorithm for detecting MR using electrocardiography (ECG); they demonstrated a promising performance of the AI algorithm for accurate MR detection. During the internal and external validation, the accuracy of MR detection was 0.816 and 0.877, respectively [16].

However, the abovementioned studies only used AI algorithms to detect MR, and there were no further qualitative studies. Recently, some studies have focused on detecting the severity of MR using automatic detection methods. Moghaddasi and Nourian developed a novel method for grading MR according to novel textural features with machine learning methods [17]. The proposed method achieved satisfactory accuracy for the detection of MR severity in normal subjects. This method is based on echocardiography videos. In their study, MR was graded into three types: mild, moderate, and severe. They did not further subdivide moderate MR into grade II and grade III. This does not reflect the severity of MR well. Studies by Uretsky et al. highlighted the accuracy and reproducibility of CMR in quantifying MR and have begun to link CMR to clinical outcomes [18]. However, in our daily practice, CMR is not widely available and is time-consuming. Moreover, in some emergency situations, CMR cannot be the first choice, and there are contraindications for it in some patients. Some studies have also pointed out that the degree of MR measured by TEE is more accurate than that measured by TTE. Militaru et al. evaluated the accuracy of MR volume quantified with 3D color Doppler TEE using new semiautomated software. The new software enabled semiautomated 3D MR flow quantification in complex MR with multiple eccentric jets and showed a satisfactory result [19]. However, TEE is operator dependent and semi-invasive, typically requiring patient sedation [20]. It is not suitable for routine examinations.

In our study, when classifying according to severity, we achieved accuracies of 0.90, 0.89, and 0.91, and when classifying according to grading, we achieved accuracies of 0.90, 0.87, 0.81, and, 0.91. Among the grading classifications, grade III has the lowest accuracy, which is mostly because the characteristics of grade III have some overlap with the characteristics of severe MR. In model verification, the unrecognized rate of grade I reached 0.04, which is probably because the VC in some images of grade I is too small to be identified. Our model also obtained better precision, recall, F1-score, Macro F1, and Micro F1. All these suggest that our model has good performance. In the process of collecting cases, the quantitative methods for MR identification in the 2017 ASE guidelines were time-consuming, and for each case, it took a few minutes to take the pictures required to obtain the results. Grade I and grade IV take less than 10 minutes to classify; however, grade II and grade III take more than 10 minutes (see Table 1). This is because when VCW ≤ 0.3 cm, VCW ≥ 0.7 cm, or some other obvious condition is present (Figure 1), it is easy to determine whether MR is mild or severe, and no further evaluation is needed. In contrast, assessing MR severity with our AI model requires a shorter amount of time, which could greatly reduce working time. This can significantly improve the work efficiency of clinicians.

In this study, we designed an experimental dataset and a validation dataset. Hospital A and hospital B are in different regions, and both hospitals are large tertiary general hospitals. This can effectively address the influence of regional differences. Three commonly used and well-known brands of ultrasound machines were used, so the accuracy and quality of performance were good. The results prove that our AI model is universally applicable and has good performance and high accuracy. More importantly, it greatly shortens the diagnosis time. Due to these advantages, this AI model has the potential to be used for diagnosis in daily clinical practice.

## 5. Conclusions

Accurate assessment of the severity of MR is crucial in clinical treatment. In this study, we chose the Mask R-CNN algorithm to qualitatively evaluate MR using color Doppler echocardiography images collected based on the 2017 ASE guidelines. This demonstrated that the model has good performance and could evaluate the severity of MR with good accuracy. Thus, with the combination of MR echocardiography images and DL, the time required to analyze cardiac-related parameters is decreased, and clinical decision-making can be expedited. This model can serve as a new tool for the evaluation of MR severity.

## Figures and Tables

**Figure 1:** Algorithm for the integration of multiple parameters of MR severity by Doppler echocardiography adapted from ASE 2017.

**Figure 2:** The workflow of LabelMe. (a) Create dataset on our local computer. (b) Perform annotation and save annotation results on each image by pressing “Save” button. (c) For each image, get a.json file, which contains for the labels created.

**Figure 3:** Example of MR contour. (a–d) The original image of MR of grade Ⅰ, grade Ⅱ, grade Ⅲ, and grade Ⅳ. (e–h) The contour map of the MR traced by the LabelMe software corresponding to (a–d).

**Figure 4:** The network architecture of Mask R-CNN.

**Figure 5:** Model performance evaluation metric and results. The abscissa axis is epoch, and the ordinate axis is loss. These four ordinates represent bbox loss, class loss, mask loss, and total loss, respectively.

**Figure 6:** Test example of assessment of MR severity. (a–d) The MR images obtained by the quantitative evaluation methods of 2017 ASE guidelines. (e–h) The grading result obtained by the Mask R-CNN algorithm. The confident scores for the four cases were 0.987, 0.986, 0.997, and 1.000, respectively.

**Figure 7:** The confusion matrix of classification results and grading results of MR. The abscissa axis is the reference results obtained through the 2017 ASE guidelines, and the ordinate axis represents the results of this research model. Unrecognized means that the model cannot recognize this MR.

**Figure 8:** Comparative histograms of precision, recall, and F1-score between classification indexes ((a) classification according to severity; (b) classification according to grading).

**Table 1:** Medical history, clinical presentation, and baseline TTE characteristics of the study patients.

	Age (Yrs)	Male	Medical history and clinical presentation						Baseline TTE characteristics					Time (minutes)
			CHD	MI	HTN	DM	TIA	NYHA≥III	LVDd, cm	LVDs, cm	LA, cm	EF, %	Reduced EF, <50%	
Mild (grade I)	61 (29-82)	126	59	14	56	41	29	19	4.3 ± 0.57	3.1 ± 0.59	3.4 ± 0.52	58 (46-67)	7	5.8 ± 4.5
Moderate (grade II)	68 (31-88)	117	102	51	82	37	27	47	4.4 ± 0.61	3.3 ± 0.58	3.5 ± 0.69	57 (44-66)	19	10.6 ± 2.7
Moderate (grade III)	71 (41-90)	121	125	62	103	38	44	91	5.1 ± 0.53	37 ± 0.65	4.2 ± 0.71	50 (36-63)	55	11.1 ± 2.4
Severe (grade IV)	73 (43-92)	135	140	71	134	47	48	135	5.5 ± 0.70	42 ± 0.87	4.5 ± 0.73	44 (30-61)	98	5.5 ± 4.4

CHD: coronary artery heart disease; MI: myocardial infarction; HTN: hypertension; DM: diabetes mellitus; TIA: transient ischemic attack; NYHA: New York Heart Association; time: the time taken to quantitatively evaluate the severity of MR according to the 2017 ASE guidelines. Values are median (interquartile range), mean ± SD, or *n* (%), unless otherwise indicated.

**Table 2:** The comparison results of Macro F1 and Micro F1 in each classification.

Classification	Macro F1	Micro F1
According to severity	0.91	0.92
According to grading	0.89	0.89

## Data Availability

The data that support the findings of this study are available from the corresponding author upon reasonable request.
